The article "The impact of antibiotic usage on the efficacy of chemoimmunotherapy is contingent on the source of tumor-reactive T cells" was published in 2017. Journal: Oncotarget.

# The impact of antibiotic usage on the efficacy of chemoimmunotherapy is contingent on the source of tumor-reactive T cells

**DOI:** 10.18632/oncotarget.22953

**Published:** 2017-12-05

**Authors:** Michal P. Kuczma, Zhi-Chun Ding, Tao Li, Tsadik Habtetsion, Tingting Chen, Zhonglin Hao, Locke Bryan, Nagendra Singh, James N. Kochenderfer, Gang Zhou

**Affiliations:** ^1^ Georgia Cancer Center, Augusta University, Augusta, Georgia, USA; ^2^ Department of Oncology and Surgery, General Hospital of Ningxia Medical University, Yinchuan, Ningxia Province, PR China; ^3^ Hematology/Oncology, Georgia Cancer Center, Augusta University, Augusta, Georgia, USA; ^4^ Department of Biochemistry and Molecular Biology, Augusta University, Augusta, Georgia, USA; ^5^ Experimental Transplantation and Immunology Branch, National Cancer Institute, Bethesda, Maryland, USA; ^6^ Current/Present address: Institute for Biomedical Sciences, Georgia State University, Atlanta, Georgia, USA

**Keywords:** antibiotics, intestinal microbiota, cyclophosphamide, chimeric antigen receptor, adoptive T-cell therapy

## Abstract

In recent years the combined use of chemotherapy and immunotherapy, collectively termed chemoimmunotherapy, has emerged as a promising treatment option for patients with cancer. Antibiotics are commonly used to reduce infection-related complications in patients undergoing chemotherapy. Intriguingly, accumulating evidence has implicated gut microbiota as a critical determinant of host antitumor immune responses, raising the question as to whether the use of broad-spectrum antibiotics would invariably diminish tumor response to chemoimmunotherapies. We investigated the impact of antibiotics on the therapeutic outcomes of cyclophosphamide (CTX) chemotherapy and adoptive T-cell therapy (ACT) where CTX was used as the host-conditioning regimen in mice. We show that antibiotic prophylaxis dampened the endogenous T cell responses elicited by CTX, and reduced the efficacy of CTX against B-cell lymphoma. In the ACT setting, antibiotics administration impaired the therapeutic effects of adoptively transferred tumor-specific CD4+ T cells in mice with implanted colorectal tumors. In contrast, long-term antibiotic exposure did not affect the efficacy of ACT using CD19-targeting chimeric antigen receptor (CAR) T cells in mice with systemic B-cell lymphoma, although it correlated with prolonged CAR expression and sustained B-cell aplasia. Our study demonstrates that chemoimmunotherapies may have variable reliance on intestinal microbiota for T cell activation and function, and thus have different sensitivities to antibiotic prophylaxis. These findings may have implications for the judicial use of antibiotics in cancer patients receiving chemoimmunotherapies.

## INTRODUCTION

In recent years the role of commensal bacteria in modulating the host antitumor immunity has become increasingly appreciated [1–3]. Accumulating evidence from animal studies demonstrated that the intestinal microbiota influences tumor response to a variety of cancer therapies, including cyclophosphamide (CTX) and platinum-based chemotherapy [4–6], a CpG oligodeoxynucleotide-based immunotherapeutic regimen [6], as well as immune checkpoint therapy such as CTLA-4 and PD-L1 blockade [7, 8]. One common feature of these therapies is that they activate the innate and adaptive immune systems, thereby eliciting endogenous immune responses that contribute to the overall antitumor efficacy [9, 10]. Disturbance of the gut microbiome by antibiotic exposure attenuates therapy-induced immune responses and diminishes the efficacy of these cancer therapies.

Adoptive T-cell therapy (ACT) has become a viable treatment option for patients with certain types of cancer [11]. Most ACT protocols involve infusion of tumor-reactive T cells following host pre-conditioning by total body irradiation (TBI) or CTX-based lymphodepletive chemotherapy [12, 13]. With the advances in cell culture methodology and T-cell engineering technology, the source of T cells has evolved from *ex vivo*-expanded tumor infiltrating lymphocytes (TILs), to T cells expressing designed tumor-specific T cell receptors (TCR) or chimeric antigen receptors (CAR)[14, 15]. Paulos et al reported in a melanoma mouse model that microbial translocation driven by TBI led to heightened dendritic cell activation which in turn augmented the function of adoptively transferred tumor-specific CD8+ T cells, and that the immunopotentiating effect of TBI was reduced in mice receiving antibiotic treatment [16]. Like TBI, the alkylating agent CTX, a chemotherapy drug often used in ACT for host pre-conditioning, can also induce microbial translocation [4, 17, 18]. These observations have led to the belief that intestinal microbes influence the effectiveness of ACT, although the impact of CTX-induced microbial translocation on ACT efficacy has not been experimentally demonstrated.

The use of CAR T cells for ACT has been an area of extensive research. So far, three generations of CAR T cells have been developed and tested in preclinical and clinical studies [19]. Among these studies, the use of the second-generation CAR T cells redirected to CD19 has manifested impressive therapeutic benefits in patients with B-cell malignancies [20], which led to FDA approval of CD19-CAR T-cell therapy for the treatment of B-cell acute lymphoblastic leukemia. A typical second-generation CAR design links an antigen-binding domain, which is usually a single-chain variable fragments (scFv) derived from a moloclonal antibody, to the T-cell signaling domain (CD3 zeta chain) coupled to the intracellular signaling domain of a costimulatory molecule such as CD28. These features facilitate robust activation of CAR T cells upon tumor encounter, and allow execution of the effector functions of CAR T cells independent of MHC restrictions. In many reported CD19-CAR T-cell therapy clinical studies, infusion of CAR T cells was preceded by CTX-based host pre-conditioning [20]. Whether CTX-induced microbial translocation contributes to the efficacy of CD19-CAR T-cell therapy is currently unclear. Moreover, the role of intestinal microbiota in ACT has particular relevance to CD19-CAR T-cell therapy. This is because patients treated with CD19-CAR T cells may experience prolonged B-cell aplasia and hypogammaglobulinemia, conditions that often require intermittent antibiotics administration and immunoglobulin replacement to reduce the risk of infection. However, whether the use of antibiotics influences the efficacy of CD19-CAR T-cell therapy has not been examined.

The current study was undertaken to investigate how antibiotics administration affects the therapeutic effects of different forms of cancer therapy involving the use of CTX as monotherapy or host pre-conditioning regimen for ACT in mouse models. We report here that antibiotic prophylaxis diminished the endogenous antitumor T cell responses elicited by CTX, impaired the efficacy of ACT using tumor-specific CD4+ T cells, but had no impact on the efficacy of ACT using CD19-CAR T cells.

## RESULTS

### Antibiotic prophylaxis impairs the antitumor effect of CTX in mice with established lymphoma

It has been reported that antibiotic treatment blunts CTX-mediated antitumor effects in a sarcoma mouse model [4]. Since CTX is widely used to treat hematologic malignancies, we asked whether antibiotics administration interferes the effectiveness of CTX against B-cell lymphoma in mice. To this end, mice were given either regular drinking water or water containing a broad-spectrum antibiotic cocktail, starting 2 weeks before inoculation of A20 B-cell lymphoma cells in the flank (Figure 1A schema). When tumor sizes reached ∼130 mm^2^, a cohort of mice in each group received one dose of CTX injection. Figure 1A shows that without treatment (no Tx), A20 tumors grew in an identical rate in mice with or without antibiotic exposure. After CTX treatment, mice on normal water or antibiotics both experienced initial tumor regression, followed by tumor regrowth (Figure 1B). Notably, relapses occurred earlier in antibiotics-treated mice than in antibiotics-naïve mice. The results support that antibiotics administration impairs the efficacy of CTX against B-cell lymphoma.

**Figure 1:** Antibiotics administration diminishes the efficacy of CTX in mice with B-cell lymphoma by attenuating CTX-elicited antitumor T cell responses **(A)** Antibiotics administration diminishes the efficacy of CTX in mice with B-cell lymphoma. The schema depicts the timeline of experimental procedures. Normal drinking water (H2O) or antibiotics-containing water (Abx) was provided to mice 2 weeks before tumor inoculation, and maintained for the duration of the experiment. A20 tumor cells were subcutaneously injected to mice on the flank. When tumor sizes reached ∼130mm^2^, mice were either left untreated (no Tx) or received CTX injection. Tumor growth curves under each condition are shown as tumor area ± SEM. Number of mice under each condition is provided. **(B)** Depletion of endogenous T cells impairs the antitumor effect of CTX. Mice with established A20 tumors were treated with CTX. Half of the mice received monoclonal antibodies to deplete CD4+ and CD8+ T cells before and after CTX treatment. Tumor growth curves are shown as tumor area ± SEM. **(C)** Antibiotics administration does not alter tumor growth rates in Rag2KO mice. Rag2KO mice were subject to the same experimental procedures describe in Figure 1A. Tumor growth curves are shown as tumor area ± SEM. ns, not significant; ^*^, *p*<0.05; ^**^, *p*<0.01.

### Antibiotics modulate CTX-mediated antitumor effect by impinging on endogenous T cells

It has been shown that the efficacy of some anticancer drugs, including CTX, is at least partially attributable to antitumor immune responses elicited by chemotherapy [21]. To determine the role of the adaptive immune system in CTX-mediated antitumor effect in our lymphoma model, tumor-bearing mice were depleted of the endogenous CD4+ and CD8+ T cells before receiving CTX treatment (Figure 1B schema). T cell-depletion led to earlier and faster tumor regrowth in mice (Figure 1B). Our results support the notion that the endogenous T cell compartment contributes to CTX-mediated tumor growth inhibition.

To determine whether provision of antibiotics affects CTX antitumor efficacy by impinging upon the host immune system, we conducted CTX treatment in the absence or presence of antibiotics in tumor-bearing immunodeficient Rag2KO mice (Figure 1C schema). Under normal water condition, CTX treatment transiently delayed tumor growth in Rag2KO mice (Figure 1C, H2O, CTX vs. H2O, no Tx); however, the process of tumor regression, which was observed in CTX-treated wild-type mice (Figure 1A), did not occur in Rag2KO mice following CTX treatment. Furthermore, antibiotics administration neither affected tumor growth rate in untreated mice, nor altered the tumor growth kinetics in CTX-treated mice. In other words, antibiotics administration, which caused faster tumor regrowth in CTX-treated wild-type mice, did not cause differences in tumor regrowth kinetics in immunodeficient mice after CTX treatment. Altogether, our data indicate that the antitumor T-cell responses elicited by CTX contribute to CTX’s overall treatment efficacy, and that the antitumor effects mediated by endogenous T cells are susceptible to modulation by the use of antibiotics.

### Antibiotics administration alters host T cell responses induced by CTX

We next examined how antibiotic treatment impacts the endogenous T-cell phenotype and functionality following chemotherapy. It appeared that antibiotics exposure reduced T cell activation induced by CTX, as reflected by decreased cell proliferation measured by Ki-67 stain in both CD4+ and CD8+ T cells, although the change in CD8+ T cells did not reach statistical significance (Figure 2A). Moreover, the fractions of effector cells (CD44+CD62L-) in both CD4+ and CD8+ T cells were reduced after antibiotic administration (Figure 2B). Furthermore, the frequencies of CD4+ and CD8+ T cells capable of producing pro-inflammatory cytokines (IFNγ^+^TNFα^+^) were significantly reduced after antibiotic treatment (Figure 2C). Of note, antibiotic exposure reduced CD40L^+^ helper CD4+ T cells as well as IL17a-producing CD4+ T cells, but had no effect on Treg cells (Figure 2D). Altogether, our data support the notion that the intestinal microbiota is a critical determinant of the host immune responses elicited by CTX, and depletion of the gut microbiome by the means of antibiotic exposure impairs T cell responses and thus diminishes the overall antitumor effect of CTX chemotherapy.

**Figure 2:** Antibiotics administration results in diminished T cell activation in CTX-treated mice Mice on normal water or antibiotics were treated with CTX. Seven days later, spleen cells were harvested for analysis. T cell proliferation status was measured by Ki67 stain **(A)**. T cell activation status was evaluated by CD44 and CD62L stain **(B)**. T cell cytokine-producing capability was evaluated by intracellular staining of IFNγ and TNFα after PMA and ionomycin stimulation **(C)**. CD4+ T cell activation marker CD40L, IL17a production, and Treg presence were also examined **(D)**. Data shown are presented as mean ± SD with 4 mice per group. ns, not significant; ^*^, *p*<0.05; ^**^, *p*<0.01.

### Antibiotics administration impairs the curative effect of adoptive CD4+ T-cell therapy in mice with implanted colorectal tumors

It has been shown that TBI-induced microbial translocation augments the efficacy of adoptively transferred tumor-specific CD8+ T cells, and that this effect is diminished after antibiotics administration [16]. CTX is widely used to condition the hosts in ACT preclinical models and clinical studies. Although CTX is known to cause microbial translocation, whether this feature contributes to ACT efficacy has not been examined. We previously established a CD4+ T cell-based ACT model system in which tumor-bearing mice receive CTX pre-conditioning followed by infusion of tumor-specific CD4+ T cells [22]. We applied this model system to mice with established HA-expressing colorectal tumor CT26HA (Figure 3 schema). As shown in Figure 3, CTX alone delayed tumor growth compared to no treatment, but this tumor-inhibiting effect was transient and tumors subsequently regrew in all mice. The combination of CTX and transfer of HA-specific CD4+ T cells (CTX+HA-CD4) led to durable complete remission in all mice 3 weeks after receiving treatment. Notably, CTX+HA-CD4 in the presence of antibiotics also led to initial tumor regression, however, the curative effect was lost in three out of five mice 3 weeks after treatment. Our data support the hypothesis that CTX-induced microbial translocation contributes to the efficacy of ACT using tumor-specific T cells.

**Figure 3:** Antibiotics administration impairs the curative effect of adoptive CD4+ T-cell therapy in a mouse colorectal tumor model The schema depicts the timeline of the experimental procedures. CT26HA tumors were subcutaneously injected to mice on the flank. A cohort of mice were provided with antibiotics-containing water during the course of experiment, starting 2 weeks before tumor inoculation. When tumor sizes reach ∼130mm^2^, mice were randomized into 3 groups to receive no treatment (no Tx), CTX only (CTX), or CTX followed by adoptive transfer of HA-specific CD4+ T cells (H2O, CTX+HA-CD4). Mice on antibiotics-containing water all received CTX and HA-CD4+ T cell transfer (Abx, CTX+HA-CD4). Tumor growth curves of each mouse under each condition are shown. The number of mice under each condition is provided.

### The use of antibiotics does not affect the efficacy of CD19-CAR T-cell therapy but influences CAR persistence and B-cell recovery

The relevance of gut microbiota to ACT using CAR T cells is currently unknown. We sought to address this using a clinically relevant mouse model of CD19-CAR T-cell therapy. Kochenderfer et al reported eradication of lymphoma and normal B cells in a preclinical model using T cell transduced with CD19-targeting CAR [23]. The viral vector MSGV-1D3-28Z-1.3 is a CD28-based second-generation CAR with the first and third ITAMs of the CD3 molecule inactivated to decrease apoptosis and increase survival of CAR-transduced T cells [23]. We used this viral vector to transduce CD45.1^+^ murine T cells for adoptive transfer. Figure 4A shows that ∼80% of T cells expressed CAR after viral transduction. The CD19 reactivity of the transduced T cells was demonstrated by the vigorous proliferation of CD19-CAR T cells in response to CD19^+^ A20 B-cell lymphoma cells but not CD19^-^ MOPC315 plasmacytoma cells during *in vitro* culture (Figure 4B). Moreover, the CD19-CAR T cells exhibited robust direct killing capability toward A20 tumor cells but not MOPC315 cells (Figure 4C).

**Figure 4:** CD19-CAR T cells exhibit direct killing activity toward B-cell lymphoma *in vitro* Total T cells isolated from the spleen of a CD45.1 BALB/c mouse were transduced with retroviral vector MSGV-1D3-28Z-1.3 to express CD19-specific CAR. **(A)** Expression of CAR in transduced T cells. To determine the expression of CAR, transduced T cells were stained with FITC-labeled polyclonal mouse anti-rat F(ab)2 antibodies to detect the 1D3 scFv, with FITC-labeled normal polyclonal mouse IgG antibodies serving as a isotype control. Percentage of CAR^+^ cells is shown. **(B)** CD19-CAR T cells proliferate in response to CD19 stimulation. CD19-CAR-transduced T cells were labeled with violet dye and incubated with equal numbers of either irradiated CD19+ A20 cells or CD19- MOPC315 cells *in vitro*. 3 days after culture, T cell proliferation reflected by dye dilution was evaluated by FACS. Number in histogram indicates % of divided cells. **(C)** CD19-CAR T cells specifically kill CD19+ B-cell lymphoma *in vitro*. Equal numbers of A20 lymphoma cells and MOPC315.GFP plasmacytoma cells were admixed. The mixed tumor cells cultured in the absence or presence of CD19-CAR-transduced T cells (CD45.1+). After overnight incubation, cells were harvested, and the composition of tumor cells were examined by flow cytometry. Histograms shown are gated on CD45.1^-^ tumor cells and the presence of A20 and MOPC315.GFP cells are distinguishable by GFP expression. Percent of A20 cells in tumor cell mixture is indicated.

Next we examined if disturbance of gut microbiota by means of antibiotic exposure affects the efficacy of CD19-CAR T-cell therapy. As depicted in Figure 5 schema, mice on normal drinking water or antibiotic cocktails were injected with A20.luci tumor cells via tail vein to establish systemic A20 tumors. Two weeks after tumor inoculation, bioluminescent imaging (BLI) was performed to document the presence of tumors in multiple organs (mostly liver and bone). Mice with comparable tumor burdens, with or without antibiotic exposure, were grouped to receive one of the three experimental conditions: no treatment, CTX only, and CTX followed by infusion of CD19-CAR T cells. We first examined the effectiveness of antibiotics in eliminating intestinal microbes. To assess the amounts of intestinal microbes, genomic DNA isolated from fresh feces were used for bacterial 16S ribosomal DNA (16S rDNA) gene amplification by qPCR as previously described [24]. Figure 5A shows that it took only ∼10 PCR cycles to enter the log phase of amplification of bacteria DNA in fecal samples collected from water-drinking mice, while more than 40 PCR cycles were needed to amplify bacteria DNA in fecal samples collected from mice under antibiotics. Furthermore, mice exposed to antibiotics exhibited enlarged cecum (Figure 5B), which is commonly seen in antibiotics-treated or germ-free mice. The results validated the efficiency of antibiotics treatment in reducing gut microbes.

**Figure 5:** The use of antibiotics does not affect the efficacy of CD19-CAR T-cell therapy but influences the persistence of CAR T cells and B cell recovery The schema depicts the timeline of the experimental procedures. Normal drinking water or antibiotics-containing water was provided to mice 2 weeks before tumor inoculation, and maintained for the duration of the experiment. A20.luci tumor cells were intravenously injected to mice. Two weeks after tumor injection, the presence of tumor in various organs was confirmed by BLI. Tumor-bearing mice were grouped and received either no treatment, CTX only, or CTX followed by infusion of CD19-CAR T cells (CD45.1^+^). The effectiveness of antibiotics in reducing intestinal microbiota was evaluated by real-time PCR detecting bacteria 16S gene in fresh feces collected on day 7. RFU-Relative Fluorescence Units **(A)**. One antibiotics-naïve mouse and one antibiotics-exposed mouse from the untreated groups were sacrificed on day 7 to examine the size of cecum as an indication of the activity of antibiotics in intestine **(B)**. Mice were monitored for survival. Overall survival of mice is shown as Kaplan-Meier survival as a function of time after CTX treatment **(C)**. The number of mice in each group is provided. **(D)** At the indicated time points, tail blood samples were collected from mice that had received CD19-CAR T cells, and examined for the presence of donor T cells (CD45.1+) and B cells (B220+CD19+) by flow cytometry. Percentages of donor cells and B cells in blood are summarized in scatter plots. **(E)** Presence of CAR in donor T cells in long-term survivors. A fraction of mice receiving CTX+CD19-CAR, in the presence of absence of antibiotics, became long-term survivors (more than 100 days after therapy). On day 145, 3 mice from each group were sacrificed and spleen cells were examined for the expression of CAR in donor T cells by Fab staining. Representative dot plots shown are gated on CD45.1+ donor T cells, and percentages of CAR+ cells in donor populations are summarized in the bar graph. The presence of B cells in spleen was evaluated by CD19 and B220 staining **(F)**. Representative dot plots are shown, and percentages of CD19^+^B220^+^ B cells in spleen are summarized in the bar graph. ns, not significant; ^*^, *p*<0.05; ^**^, *p*<0.01; ^***^, *p*<0.001.

We used animal survival as a functional readout to evaluate the physiological impact of antibiotics administration. All untreated mice died within 20 days (34 days after tumor inoculation), whether or not antibiotics were provided (Figure 5C, no Tx groups). CTX treatment prolonged mouse survival, however, the efficacy of CTX was impaired by antibiotics administration, as evidenced by reduction in the median survival from 38 days to 22 days (Figure 5A, H2O, CTX versus Abx, CTX). For CD19-CAR T-cell therapy, in which CD19-CAR T cells were infused to mice after CTX-preconditioning, the survival rate in mice on normal drinking water was not statistically different from that in mice on antibiotics (Figure 5C, H2O, CTX+CD19CAR versus Abx, CTX+CD19CAR).

We collected peripheral blood from a cohort of mice at different time points to examine the impact of antibiotics administration on the presence of the donor T cells, as well as the occurrence of B-cell aplasia. Figure 5D shows that donor T cell frequencies were mostly comparable in antibiotics-treated mice compared to antibiotics-naïve mice at the time points examined. Moreover, B-cell aplasia was evident in both antibiotics-naïve and antibiotics-treated mice soon after CD19 CAR T therapy (day 10). Notably, B cells started to re-emerge in antibiotics-naïve mice at later times (2 out of 5 on day 20, 4 out 5 on day 35), whereas B-cell aplasia persisted in antibiotics-treated mice. After CD19-CAR T-cell therapy, a fraction of mice, with or without antibiotic exposure, achieved long-term survival (more than 100 days after therapy), and remained tumor-free as reflected by lack of tumor signal measured by BLI (data not shown). We sacrificed 3 mice from each group to analyze the presence of CAR+ donor T cells and host B cells in spleens. Figure 5E shows that among the CD45.1^+^ donor cells found in spleens, CAR-expressing cells were nearly absent in antibiotics-naïve mice but easily detectable in antibiotics-treated mice. CD19+ B cells were fully recovered in the spleens of antibiotics-naïve mice but absent in antibiotics-treated mice (Figure 5F), showing an inverse correlation with the presence of CAR+ T cells. In sum, our data indicate that antibiotics administration has no impact on the efficacy of CD19-CAR T-cell therapy, but affects the persistence of CAR-expressing donor T cells and the duration of B-cell aplasia.

## DISCUSSION

CTX is a component of frontline therapies for many types of cancer. Here we show that the endogenous T cell responses elicited by CTX contributed to the overall efficacy of CTX against A20 B-cell lymphoma. Moreover, antibiotics administration resulted in reduced antitumor effect of CTX, and was associated with diminished endogenous T-cell responses. Our data are consistent with the results of two recent studies reporting that intestinal microbiota modulates the antitumor immune effects of CTX in a sarcoma mouse model [4, 5], suggesting the generality of reliance of CTX chemotherapy on gut bacteria to provoke antitumor immune responses.

CTX is also widely used as a host-conditioning regimen in ACT. Its immunopotentiating effects are attributed to its ability to enhance tumor antigen presentation by inducing immunogenic cell death, reduce immunosuppression by depleting Treg cells, and promote donor T cell expansion and survival by creating space and removing “cytokine sinks” as a result of lymphopenia [25, 26]. In the clinic, the sources of T cells used for ACT include patient-derived *ex vivo*-expanded TILs, selected tumor-reactive T cell clones, and T cells genetically modified to express tumor-specific TCRs or CARs [14]. In the current study, we employed two types of T cells, tumor-specific CD4+ T cells or CD19-CAR T cells, for adoptive transfer following CTX-mediated host-conditioning. The dose of CTX we used (150 mg/kg) causes transient lymphodepletion in mice and is widely used in animal ACT studies. We used one dose of CTX throughout our study so that the impact of CTX on the host is comparable among different tumor models. In a colorectal tumor model, tumor-specific CD4+ T cells derived from TCR transgenic (TCR-Tg) mice were used, modeling the clinical use of selected tumor-reactive T cell clones or T cells engineered to express tumor-specific TCRs. We show that antibiotics administration had detrimental effect on the efficacy of ACT using tumor-specific CD4+ T cells. Our results echo the study by Paulos et al showing that in a melanoma model antibiotics administration reduced the efficacy of tumor-specific TCR-Tg CD8+ T cells transferred after TBI-mediated host-conditioning [16]. In contrast, we show that in mice pre-conditioned by CTX, the therapeutic efficacy of CD19-CAR T cells against systemic B-cell lymphoma was insensitive to antibiotics.

The different sensitivity of TCR-Tg T cells and CD19-CAR T cells to antibiotics reflects differential dependence of these T cells on intestinal microbiota for executing their effector functions. It has been shown that TBI-induced microbial translocation represents one important mechanism by which TBI enhances the efficacy of ACT [16]. Mechanistically, TBI-induced microbial translocation leads to heightened DC activation which subsequently augments the function of adoptively transferred tumor-specific CD8+ T cells. CTX is also known to cause translocation of bacteria across the intestinal epithelium [4, 17, 18]. Thus, it is conceivable that CTX may resemble TBI in augmenting the function of adoptively transferred tumor-specific T cells, i.e. TCR-Tg T cells, through mechanisms triggered by microbial translocation and DC activation. Indeed, we found that the presence of antibiotics in cell culture did not affect T cell expansion and cytokine production during *in vitro* antigenic stimulation (data not shown), suggesting that antibiotics may indirectly impact T cell function *in vivo* through modulating DC activation. The loss of sensitivity to antibiotics by CD19-CAR T cells indicates that CTX-induced microbial translocation does not impact the function of CD19-CAR T cells. This phenomenon may be attributable to the unique feature of CAR T cells. CD19-CAR-transduced T cells are genetically modified such that the tumor antigen-binding domain (scFv) is directly linked to the costimulatory and CD3zeta signaling domains. Thus, CD19-CAR T cells are equipped to exert effector functions instantly upon tumor encounter, without the need to be reactivated by DCs following adoptive transfer.

Although antibiotics administration did not affect the antitumor effects of CD19-CAR T-cells, it had profound impact on the persistence of CAR and B-cell recovery in the A20 lymphoma model. We show that durable complete remission was achieved in ∼40% of mice with disseminated B-cell lymphoma after CD19-CAR T-cell therapy. However, in the mice achieving complete remission, the donor T cells lost CAR expression and the level of B cells (CD19+B220+) rebounded to the level of normal mice. Our data is reminiscent of an earlier report by Cheadle et al showing the occurrence of tumor eradication, B-cell recovery and CAR-T cell disappearance in mice receiving T cells transduced with a first-generation CD19-CAR vector [27]. Several CD28-based second-generation CD19 CAR-T therapy models have been reported in literature. Although the CD19-CAR vectors used in these studies all adopted 1D3 scFv for CD19-targeting, they had differences in other elements of CAR structure that may influence CAR-T cell function, including signal peptide, linker sequences, length of the hinge domain, mutations in CD3ζ ITAMs, and the origin of species of CD28 and CD3ζ molecules (human versus mouse). Although these studies all demonstrated high response rates and curative outcomes in mice of different strains implanted with various CD19-expressing tumor cell lines, there were variations in terms of CAR T cell persistence and duration of B-cell aplasia [28, 29]. These variations may stem from different combinations of multiple factors, including different CAR designs, mouse strains, tumor types, and host preconditioning regimen (CTX versus TBI). Using a clinically relevant CD19-CAR model system, our study provides the first indication that prophylactic antibiotic usage is associated with prolonged CAR presence in donor T cells and sustained B-cell aplasia. The exact mechanisms underlying this phenomenon are currently unknown. We hypothesize that the marked reduction of intestinal microbiota by antibiotics may inhibit or delay B cell repopulation after lymphodepletion, allowing the infused CD19-CAR T cells to effectively eliminate any nascent CD19+ B cells. Consequently, B-cell aplasia is maintained and CD19-CAR T cells persist in antibiotics-treated mice. In contrast, in antibiotics-naïve mice CD19-CAR T cells have to constantly encounter a large number of B cells rebounding after chemotherapy and may undergo apoptosis due to activation-induced cell death (AICD), eventually leading to B-cell recovery and CAR T cell disappearance. These possibilities will be investigated in future studies.

The use of antibiotics has important clinical implications for chemotherapy. Infections pose a serious threat to cancer patients undergoing chemotherapy, accounting for much of the morbidity and mortality [30–32]. The use of prophylactic antibiotics in combination with chemotherapy to prevent infection-related complications is common. With particular relevance to CD19-CAR T-cell therapy, patients treated with CD19-CAR T cells may experience prolonged B-cell aplasia and hypogammaglobulinemia [33, 34], conditions that often require intermittent antibiotics administration and immunoglobulin replacement to reduce the risk of infection [35, 36]. Our study, together with others, suggests caution in antibiotic usage in therapies whose efficacies partly rely on intestinal microbial translocation, such as CTX-based chemotherapy and ACT using T cells with natural or engineered tumor-specific TCRs. In fact, the findings from animal studies are supported by emerging clinical data, which implicate a negative correlation between antibiotics usage and the antitumor activity of CTX in patients with chronic lymphocytic leukemia (CLL) [37]. On the other hand, our data imply that the robust antitumor effects exerted by CD19-CAR T cells are unlikely to be affected by intermittent short-term antibiotics administration, alleviating the concern about interference of treatment efficacy by antibiotics.

In summary, we show in mice that antibiotic prophylaxis diminished the therapeutic effect of CTX against B-cell lymphoma by attenuating the endogenous T cell responses elicited by CTX. In the ACT setting where exogenous tumor-reactive T cells were infused to CTX-conditioned mice, antibiotics administration reduced the efficacy of tumor-specific CD4+ T cells in a colorectal tumor model. In contrast, long-term antibiotic exposure had no impact on the effectiveness of ACT using CD19-CAR T cells in the treatment of systemic lymphoma, although it influenced the persistence of CAR expression and the duration of B-cell aplasia. Our study suggests that the reliance of chemoimmunotherapies on intestinal microbiota to initiate and augment antitumor immune responses may vary depending on the nature of antigen-recognition and mechanism of action of the tumor-reactive T cells. Our findings may have implications for antibiotic usage in cancer patients receiving chemoimmunotherapies.

## MATERIALS AND METHODS

### Mice

Female BALB/c (CD45.2) mice (4–6 wk old) were purchased from Charles River (Frederick, MD). HA-TCR transgenic (Tg) mice on a BALB/c background expressing an αβ TCR specific for amino acids 110–120 from influenza hemagglutinin (HA) presented by MHC class II (MHC-II) molecule I-E^d^ were described previously [22]. CD45.1 mice were purchased from The Jackson Laboratory (Bar Harbor, ME). Rag2^-/-^ mice on BALB/c background were purchased from Taconic. All animal experiments were approved by the Institutional Animal Care and Use Committee of the Augusta University.

### Antibodies and reagents

The following fluorochrome-conjugated antibodies were used for flow cytometry: anti-mouse CD44-FITC (IM7), CD11C-APC (N418), IFNγ-APC (XMG1.2), B220-PE (RA3-6B2), CD19-FITC (1D3), CD62L-PE (MEL-14), CD8-PE (53–6.7), CD40L-PE (MR1), TNFα-PE (MP6-XT22), CD4-APC/Cy7 (RM4-5) and control IgG mAbs were purchased from Biolegend. Ki67-FITC staining set was purchased from BD. Foxp3-APC staining kit was purchased from eBiosciences. Cell Proliferation Dye eFluor™ 450 were purchased from Invitrogen. Cyclophosphamide (CTX) was from MP Biomedicals and was intraperitoneally injected to mice at 150 mg/kg. Retronectin was from Takara and was used for coating of non-treated plates (Corning) at 12 μg/ml. For T cell depletion, anti-CD4 (clone GK1.5) and anti-CD8 (clone 2.43) antibodies, both from BioXCell, were injected i.p. at 100 μg each per mouse 2 days before CTX and were administered once a week thereafter for a total of 4 injections.

### Antibiotics treatment

The antibiotics cocktail containing ciprofloxacin (TCI, Portland, Oregon, 0.15 g/liter), gentamicin (0.2 g/liter), bacitracin (1g/liter) and streptomycin (2 g/liter) (Thermo-Fisher, Waltham, MA) in drinking water was given to mice *ad libitum*.

### Tumor cell lines, animal tumor models and adoptive cell transfer

Murine B-cell lymphoma cell line A20 were obtained from ATCC. A20 cells expressing luciferase (A20.luci), HA-expressing colorectal carcinoma (CT26HA) and plasmacytoma (MOPC315.GFP) cell lines were described previously [38–40]. Tumor cells were subcutaneously (4 × 10^6^) or intravenously (1 × 10^6^) injected to mice. For subcutaneous tumor models (A20 and CT26HA), tumor growth was monitored by caliper measurement of the tumor area every other day and was expressed in square millimeters by product of two perpendicular dimensions. For systemic B-cell lymphoma model (A20.luci), tumor burden was measured by bioluminescence imaging (BLI) using an Ami-x instrument (Spectral Instruments) after intraperitoneal injection of luciferin (Thermo; 150 mg/kg in PBS). For CD19-CAR T cell transfer, a total of 5 × 10^6^ transduced T cells per mouse were injected. Antibiotics were administered to mice in drinking water two weeks before inoculation of tumor cells.

### Cell preparation and flow cytometry analysis

Single cell suspensions were prepared from mice tail blood or spleen for flow cytometry analysis. For surface molecule detection, 1 × 10^6^ cells were stained with pre-titrated monoclonal Abs for 20 minutes at room temperature in the dark. Cells were washed twice with PBS and used for analysis. For detection of CD19-CAR expression in transduced T cells, Fluorescein isothiocyanate (FITC)–labeled polyclonal mouse anti–rat-F(ab)_2_ antibodies (Jackson ImmunoResearch Laboratories) were used to detect the 1D3 scFv; FITC–labeled normal polyclonal mouse IgG antibodies (Jackson ImmunoResearch Laboratories) served as an isotype control. For Foxp3 staining, Foxp3 staining kit (eBioscience) was used following manufacturer’s instruction. For intracellular cytokine staining, T cells were stimulated with PMA/ionomycin in the presence of GolgiStop for 4 hours at 37°C. Cells were harvested and stained for IFN-γ, TNF-α and IL17a using the Cytokine fix/perm kit (BD). Data were acquired using LSR II instrument (BD Biosciences). All data were analyzed using FlowJo software (version 9.7.6; Tree Star).

### Isolation and detection of microbial DNA

Microbial DNA was isolated from fresh feces with Qiagen Stool Mini kit. Mouse feces were collected directly to sterile 1.5 ml tubes, snap frozen on dry ice/ethanol and stored at -80°C until use. For DNA isolation, 150 mg of each fecal sample was processed according to manufacturer’s protocol. Each DNA was eluted with 100 μl of elution buffer and stored at -20°C until use. The abundance of intestinal bacteria was evaluated using universal total bacterial 16S ribosomal DNA primers (forward primer 5’-ACTCCTACGGGAGGCAGCAGT-3’ and reverse primer 5’-GTATTACCGCGGCTGCTGGCAC-3’) that detect the common fragment found in bacterial genomic DNA.

### Virus preparation and T cell transduction

Detailed protocol for T cell viral transduction was previously described [23]. Briefly, T cells were purified from spleens of BALB/c mice on CD45.1 background using the EasySep™ Mouse T Cell Isolation Kit (STEMCELL Technologies). T cells were cultured in the presence of hIL2 (30U/ml; NCI) and stimulated with CD3/CD28 activation Dynal beads (Invitrogen) according to manufacturer’s instruction. Activated T cells were transduced twice in two consecutive days with retroviral supernatant using retronectin. One day after the last viral transduction, Dynal beads were removed and cells were washed with PBS for *in vitro* analysis or adoptive transfer. The transduction efficiency was evaluated by staining T cells with FITC-labeled mouse anti-rat Fab antibodies or isotype control.

### Statistical analysis

Data are presented as the mean values ± SD or Kaplan-Meier survival plots. The significance of differences between samples or groups of mice was determined using paired, one-tailed Student t test. Differences between samples with p values ≤0.05 were considered significant. Statistical analysis was done using Prism 5.0 (GraphPad).

## Abbreviations

CTX: cyclophosphamide
ACT: adoptive T-cell therapy
CAR: chimeric antigen receptor
TBI: total body irradiation
scFv: single chain variable fragment
BLI: bioluminescent imaging

## References

[1] Nelson MH, Diven MA, Huff LW, Paulos CM (2015). Harnessing the microbiome to enhance cancer immunotherapy. J Immunol Res.

[2] Zitvogel L, Ayyoub M, Routy B, Kroemer G (2016). Microbiome and anticancer immunosurveillance. Cell.

[3] Perez-Chanona E, Trinchieri G (2016). The role of microbiota in cancer therapy. Curr Opin Immunol.

[4] Viaud S, Saccheri F, Mignot G, Yamazaki T, Daillere R, Hannani D, Enot DP, Pfirschke C, Engblom C, Pittet MJ, Schlitzer A, Ginhoux F, Apetoh L (2013). The intestinal microbiota modulates the anticancer immune effects of cyclophosphamide. Science.

[5] Daillere R, Vetizou M, Waldschmitt N, Yamazaki T, Isnard C, Poirier-Colame V, Duong CP, Flament C, Lepage P, Roberti MP, Routy B, Jacquelot N, Apetoh L (2016). Enterococcus hirae and Barnesiella intestinihominis facilitate cyclophosphamide-induced therapeutic immunomodulatory effects. Immunity.

[6] Iida N, Dzutsev A, Stewart CA, Smith L, Bouladoux N, Weingarten RA, Molina DA, Salcedo R, Back T, Cramer S, Dai RM, Kiu H, Cardone M (2013). Commensal bacteria control cancer response to therapy by modulating the tumor microenvironment. Science.

[7] Vetizou M, Pitt JM, Daillere R, Lepage P, Waldschmitt N, Flament C, Rusakiewicz S, Routy B, Roberti MP, Duong CP, Poirier-Colame V, Roux A, Becharef S (2015). Anticancer immunotherapy by CTLA-4 blockade relies on the gut microbiota. Science.

[8] Sivan A, Corrales L, Hubert N, Williams JB, Aquino-Michaels K, Earley ZM, Benyamin FW, Lei YM, Jabri B, Alegre ML, Chang EB, Gajewski TF (2015). Commensal Bifidobacterium promotes antitumor immunity and facilitates anti-PD-L1 efficacy. Science.

[9] Goldszmid RS, Dzutsev A, Viaud S, Zitvogel L, Restifo NP, Trinchieri G (2015). Microbiota modulation of myeloid cells in cancer therapy. Cancer Immunol Res.

[10] Honda K, Littman DR (2016). The microbiota in adaptive immune homeostasis and disease. Nature.

[11] Rosenberg SA, Restifo NP (2015). Adoptive cell transfer as personalized immunotherapy for human cancer. Science.

[12] Muranski P, Boni A, Wrzesinski C, Citrin DE, Rosenberg SA, Childs R, Restifo NP (2006). Increased intensity lymphodepletion and adoptive immunotherapy—how far can we go?. Nat Clin Pract Oncol.

[13] Dudley ME, Yang JC, Sherry R, Hughes MS, Royal R, Kammula U, Robbins PF, Huang J, Citrin DE, Leitman SF, Wunderlich J, Restifo NP, Thomasian A (2008). Adoptive cell therapy for patients with metastatic melanoma: evaluation of intensive myeloablative chemoradiation preparative regimens. J Clin Oncol.

[14] Feldman SA, Assadipour Y, Kriley I, Goff SL, Rosenberg SA (2015). Adoptive cell therapy—tumor-infiltrating lymphocytes, T-cell receptors, and chimeric antigen receptors. Semin Oncol.

[15] Barrett DM, Grupp SA, June CH (2015). Chimeric antigen receptor- and TCR-modified T cells enter main street and wall street. J Immunol.

[16] Paulos CM, Wrzesinski C, Kaiser A, Hinrichs CS, Chieppa M, Cassard L, Palmer DC, Boni A, Muranski P, Yu Z, Gattinoni L, Antony PA, Rosenberg SA (2007). Microbial translocation augments the function of adoptively transferred self/tumor-specific CD8+ T cells via TLR4 signaling. J Clin Invest.

[17] Yang J, Liu KX, Qu JM, Wang XD (2013). The changes induced by cyclophosphamide in intestinal barrier and microflora in mice. Eur J Pharmacol.

[18] Xu X, Zhang X (2015). Effects of cyclophosphamide on immune system and gut microbiota in mice. Microbiol Res.

[19] Sadelain M, Brentjens R, Riviere I (2013). The basic principles of chimeric antigen receptor design. Cancer Discov.

[20] Sadelain M (2015). CAR therapy: the CD19 paradigm. J Clin Invest.

[21] Zitvogel L, Apetoh L, Ghiringhelli F, Kroemer G (2008). Immunological aspects of cancer chemotherapy. Nat Rev Immunol.

[22] Ding ZC, Blazar BR, Mellor AL, Munn DH, Zhou G (2010). Chemotherapy rescues tumor-driven aberrant CD4+ T-cell differentiation and restores an activated polyfunctional helper phenotype. Blood.

[23] Kochenderfer JN, Yu Z, Frasheri D, Restifo NP, Rosenberg SA (2010). Adoptive transfer of syngeneic T cells transduced with a chimeric antigen receptor that recognizes murine CD19 can eradicate lymphoma and normal B cells. Blood.

[24] Sivaprakasam S, Gurav A, Paschall AV, Coe GL, Chaudhary K, Cai Y, Kolhe R, Martin P, Browning D, Huang L, Shi H, Sifuentes H, Vijay-Kumar M (2016). An essential role of Ffar2 (Gpr43) in dietary fibre-mediated promotion of healthy composition of gut microbiota and suppression of intestinal carcinogenesis. Oncogenesis.

[25] Sistigu A, Viaud S, Chaput N, Bracci L, Proietti E, Zitvogel L (2011). Immunomodulatory effects of cyclophosphamide and implementations for vaccine design. Semin Immunopathol.

[26] Proietti E, Moschella F, Capone I, Belardelli F (2012). Exploitation of the propulsive force of chemotherapy for improving the response to cancer immunotherapy. Mol Oncol.

[27] Cheadle EJ, Hawkins RE, Batha H, O'Neill AL, Dovedi SJ, Gilham DE (2010). Natural expression of the CD19 antigen impacts the long-term engraftment but not antitumor activity of CD19-specific engineered T cells. J Immunol.

[28] Davila ML, Kloss CC, Gunset G, Sadelain M (2013). CD19 CAR-targeted T cells induce long-term remission and B Cell Aplasia in an immunocompetent mouse model of B cell acute lymphoblastic leukemia. PLoS One.

[29] Cheadle EJ, Sheard V, Rothwell DG, Bridgeman JS, Ashton G, Hanson V, Mansoor AW, Hawkins RE, Gilham DE (2014). Differential role of Th1 and Th2 cytokines in autotoxicity driven by CD19-specific second-generation chimeric antigen receptor T cells in a mouse model. J Immunol.

[30] van Vliet MJ, Tissing WJ, Dun CA, Meessen NE, Kamps WA, de Bont ES, Harmsen HJ (2009). Chemotherapy treatment in pediatric patients with acute myeloid leukemia receiving antimicrobial prophylaxis leads to a relative increase of colonization with potentially pathogenic bacteria in the gut. Clin Infect Dis.

[31] van Vliet MJ, Harmsen HJ, de Bont ES, Tissing WJ (2010). The role of intestinal microbiota in the development and severity of chemotherapy-induced mucositis. PLoS Pathog.

[32] Hubel K, Hegener K, Schnell R, Mansmann G, Oberhauser F, Staib P, Diehl V, Engert A (1999). Suppressed neutrophil function as a risk factor for severe infection after cytotoxic chemotherapy in patients with acute nonlymphocytic leukemia. Ann Hematol.

[33] Kochenderfer JN, Wilson WH, Janik JE, Dudley ME, Stetler-Stevenson M, Feldman SA, Maric I, Raffeld M, Nathan DA, Lanier BJ, Morgan RA, Rosenberg SA (2010). Eradication of B-lineage cells and regression of lymphoma in a patient treated with autologous T cells genetically engineered to recognize CD19. Blood.

[34] Kalos M, Levine BL, Porter DL, Katz S, Grupp SA, Bagg A, June CH (2011). T cells with chimeric antigen receptors have potent antitumor effects and can establish memory in patients with advanced Leukemia. Sci Transl Med.

[35] Namuduri M, Brentjens RJ (2016). Medical management of side effects related to CAR T cell therapy in hematologic malignancies. Expert Rev Hematol.

[36] Lee DW, Gardner R, Porter DL, Louis CU, Ahmed N, Jensen M, Grupp SA, Mackall CL (2014). Current concepts in the diagnosis and management of cytokine release syndrome. Blood.

[37] Pflug N, Kluth S, Vehreschild JJ, Bahlo J, Tacke D, Biehl L, Eichhorst B, Fischer K, Cramer P, Fink AM, von Bergwelt-Baildon M, Stilgenbauer S, Hallek M (2016). Efficacy of antineoplastic treatment is associated with the use of antibiotics that modulate intestinal microbiota. Oncoimmunology.

[38] Ding ZC, Liu C, Cao Y, Habtetsion T, Kuczma M, Pi W, Kong H, Cacan E, Greer SF, Cui Y, Blazar BR, Munn DH, Zhou G (2016). IL-7 signaling imparts polyfunctionality and stemness potential to CD4(+) T cells. Oncoimmunology.

[39] Lu X, Ding Z, Cao Y, Liu C, Habtetsion T, Yu M, Lemos H, Salman H, Xu H, Mellor AL, Zhou G (2015). Alkylating agent melphalan augments the efficacy of adoptive immunotherapy using tumor-specific CD4+ T Cells. J Immunol.

[40] Riedel SS, Mottok A, Brede C, Bauerlein CA, Jordan Garrote AL, Ritz M, Mattenheimer K, Rosenwald A, Einsele H, Bogen B, Beilhack A (2012). Non-invasive imaging provides spatiotemporal information on disease progression and response to therapy in a murine model of multiple myeloma. PLoS One.

